The article "Ligustrazine inhibits the proliferation and migration of ovarian cancer cells via regulating miR-211" was retracted in 2024. Reasons: plagiarized images; overlap with other authors' work; signs of a paper mill; concerns about the images.

# Ligustrazine inhibits the proliferation and migration of ovarian cancer cells via regulating miR-211

**DOI:** 10.1042/BSR20200199

**Published:** 2021-01-05

**Authors:** Hairong Zhang, Shichao Ding, Lei Xia

**Affiliations:** 1 Department of Obstetrics and Gynecology, Shandong Provincial Third Hospital, Cheeloo College of Medicine, Shandong University, Jinan 250031, China; 2 Department of Internal Medicine, The Third Affiliated Hospital of Shandong First Medical University, Jinan 250031, China; 3 Department of Internal Medicine, Affiliated Hospital of Shandong Academy of Medical Sciences, Jinan 250031, China; 4 Department of Pathology, Shandong University of Traditional Chinese Medicine, Jinan 250355, China

**Keywords:** EMT, LSZ, miR-211, SK-OV-3

## Abstract

Ovarian cancer (OC) is a commonly diagnosed female cancer. Ligustrazine (LSZ), a natural compound, has been reported to exert anti-cancer activity, although the mechanisms underlying the anti-cancer effects are not clear. The present study investigated the impact of LSZ on cell proliferation and migration by regulating microRNA-211 (miR-211) expression using the human ovarian cancer SK-OV-3 and OVCAR-3 cell lines. OC cells were treated with 0, 0.5, 1, and 2 mM LSZ, and quantitative real-time PCR was utilized to measure miR-211 levels in SK-OV-3 and OVCAR-3 cells with different treatment. Moreover, to further confirm the roles of miR-211 in LSZ induced anti-tumor effects, miR-211 expression was inhibited by transfection of miR-211 inhibitors in SK-OV-3 cells. Cell proliferation of transfected cells was evaluated using the CCK-8 and colony formation assay. The scratch assay was employed to assess cell migration and transwell assay was performed for evaluating the cell invasion. Protein levels of epithelial–mesenchymal transition (EMT) markers were determined by Western blotting. We found that LSZ inhibited the viability, proliferation, migration and invasion ability of SK-OV-3 and OVCAR-3 cells in a dose-dependent manner; moreover, LSZ could significantly increase the expression of miR-211 in both SK-OV-3 and OVCAR-3, and knockdown of miR-211 in SK-OV-3 cells partially abrogated the anti-tumor behavior of LSZ by promoting the viability, proliferation, migration, invasion and EMT of SK-OV-3 cells. Thus, we found that LSZ can inhibit the proliferation and migration of OC cells via regulating miR-211. Our study suggests that LSZ might be a potential and effective treatment for OC.

## Introduction

Ovarian cancer (OC) is a commonly diagnosed female cancer worldwide [1–3]. Like most types of cancer, OC lacks clinical symptoms at its early stages, therefore, most patients have proceeded to the advanced stage at the time of diagnosis [4–6]. Moreover, the pathogenesis of OC remains unclear, and there are no specific therapies for OC, leading to an adverse prognosis of the disease [7–9]. Thus, it is of great importance to develop new therapeutic strategies to improve the therapeutic efficacy of OC and to increase the 5-year survival rate of OC patients.

The article "Ligustrazine inhibits the proliferation and migration of ovarian cancer cells via regulating miR-211" was retracted in 2024. Reasons: plagiarized images; overlap with other authors' work; signs of a paper mill; concerns about the images.

In recent years, the role of traditional medicines as alternative therapeutic methods for the treatment of cancers has been evaluated in many studies [10,11]. Ligustrazine (LSZ) is an active component used in Traditional Chinese Medicine extracted from the rhizome of *Ligusticum wallichii*. Previous studies have suggested that LSZ can exert anti-inflammatory, anti-fibrotic, and anti-oxidant activities. In some recent studies, a tumor suppressive activity of LSZ has been described for several cancers, including lung cancer, gastric cancer, breast cancer, and melanoma [10–16].

MicroRNAs (miRNAs) are a class of single-stranded RNAs. Unlike messenger RNAs (mRNA), miRNAs are not translated into a protein, although they can bind to the 3′-UTR of their target mRNAs and can epigenetically inhibit the expression of their target genes [17,18]. Over the past few decades, the roles of miRNAs in different types of cancers, including OC, have been extensively investigated [19,20], and several miRNAs have been identified as potential therapeutic targets for the treatment of OC [21–24].

LSZ has been reported to exert its anti-tumor effects by inhibiting the growth, migration, and epithelial–mesenchymal transition (EMT) of different types of cancer cells, including OC [10,25,26]. On the other hand, LSZ has been reported to regulate cellular activities through its effects on the expression of several miRNAs [26,27]. MicroRNA-211 (MiR-211) is considered a tumor suppressor in the pathogenesis of OC, however, whether LSZ regulates the expression of miR-211, and thus contributes to its anti-tumor activity in the pathogenesis of OC remains to be explored. In the present study, our aim was to explore the effects of LSZ on the migration, invasion, and EMT of OC cells. The roles played by miR-211 during these processes was also investigated.

## Materials and methods

### Cell lines and treatment

The human OC line SK-OV-3 and OVCAR-3 were purchased from ATCC (Manassas, VA, U.S.A.). Cells were cultured in RPMI-1640 medium (Gibco, CA, U.S.A.) containing 10% fetal bovine serum (Gibco), with 100 U/ml penicillin and 100 μg/ml streptomycin (Gibco). Cells were cultured in an incubator at 37°C, and supplied with 5% CO_2_. To determine the effects of LSZ on the behavior of SK-OV-3 cells, cells were treated with 0, 0.5, 1, and 2 mM LSZ at different time points (Sigma–Aldrich Corp., St. Louis, MO, U.S.A.).

The article "Ligustrazine inhibits the proliferation and migration of ovarian cancer cells via regulating miR-211" was retracted in 2024. Reasons: plagiarized images; overlap with other authors' work; signs of a paper mill; concerns about the images.

### Transfection

To explore the role of miR-211 in LSZ-induced effects on SK-OV-3 and OVCAR-3 cells, cells were seeded on to 24-well plates and randomly divided into the following groups: blank control group, LSZ group (cells treated with 1 mM LSZ), LSZ+miR-211 inhibitor group (cells treated with 1 mM LSZ), and the ginsenoside-Rg3+ HOTAIR control group. Cells were transfected with the miR-211 inhibitor in a 2.5 µl volume of Lipofectamine 2000 (Invitrogen, U.S.A.). Experiments were performed in triplicate.

### CCK-8 cell viability assay

Cell viability was determined using the CCK-8 cell viability assay. Briefly, cells were seeded on to a 96-well plate and the CCK-8 solution (purchased from Beyotime, Shanghai, China) was added to the wells (10 μl/well) and incubated at 37°C for 2 h. Next, the optical density (OD) value was measured at the wavelength of 450 nm using a microplate reader (Bio-Rad, Hercules, CA, U.S.A.) to evaluate the viability of the cells at different treatment concentrations.

### Colony formation assay

Colony formation assay was performed to determine the proliferation ability of SK-OV-3 and OVCAR-3 cells. Briefly, cells were cultured for 10 days, fixed in methanol, and then stained by Crystal Violet (0.1%). Colonies (diameter ≥ 100 μm) were counted microscopically.

### Quantitative real-time polymerase chain reaction

The expression of miR-211 was determined using quantitative real-time polymerase chain reaction (qRT-PCR). RNeasy Mini Kit (Qiagen, Germany) was utilized to isolate RNA according to the manufacturer’s protocol and the concentration of RNA was identified by a spectrophotometer Nanodrop 2000 (Thermo Fisher Scientific, U.S.A.). The M-MLV was applied to synthesize cDNA through reverse transcription. PrimeScript™ RT-PCR Kit (TaKaRa, Japan) was used for RT-PCR. For cDNA synthesis, samples were incubated at 43°C for 30 min, 97°C for 5 min, and 5°C for 5 min. The thermal cycling parameters were as follows: 95°C for 5 min followed by 40 cycles of 95°C for 30 s, 59°C for 30 s, 72°C for 30 s. GAPDH was regarded as an internal control. Each experiment was performed in triplicate. The abundance of gene expression was determined by 2^−ΔΔ*C*_t_^ relative quantification [18].

### Western blotting

Western blotting was used to assess protein expression. Cells were lysed in RIPA buffer (Thermo Fisher Scientific, U.S.A.) and the total protein concentration was verified by the BCA Kit (Thermo Fisher Scientific, U.S.A.). A total of 20 µg of proteins were separated by gel electrophoresis (15% SDS/PAGE) and then transferred to PVDF membrane (Millipore, Netherlands). The membrane was blocked with 5% skimmed milk for 2 h. Subsequently, the primary antibodies were incubated for 1 h at room temperature. Next, the membrane was incubated with the relative secondary antibody (ab6721, 1:2000, Abcam, U.S.A.) conjugated with HRP for 45 min at room temperature. Then, the ECL Western Blotting Kit (Santa Cruz Biotechnology, Inc.) was used for membrane staining and the results were analyzed with ImageJ software. Each experiment was performed in triplicate.

The article "Ligustrazine inhibits the proliferation and migration of ovarian cancer cells via regulating miR-211" was retracted in 2024. Reasons: plagiarized images; overlap with other authors' work; signs of a paper mill; concerns about the images.

### Scratch-wound healing assay

The scratch-wound healing assay was employed to evaluate the migration and invasion ability of SK-OV-3 and OVCAR-3 cells. Cells were seeded into 96-well plates and a monolayer cell culture was obtained. Next, a new 1-ml pipette tip was used to generate a scratch across the center of the wells. Therefore, the width of the scratch was defined by the outer diameter of the tip. The cells were then incubated at 37°C with 5% CO_2_ for 72 h. The migrated cells were captured by microscope (Olympus, Tokyo, Japan).

### Transwell cell invasion assay

SK-OV-3 and OVCAR-3 cells were seeded on to the upper chamber of the transwell pre-coated with Matrigel (BD Biosciences) and incubated for 24 h. Next, the invaded cells were fixed by paraformaldehyde (4%) and then stained by 0.1% Crystal Violet and imaged by a microscope.

### Statistical analysis

All data are presented as the mean ± standard deviation (SD) and were analyzed using GraphPad Prism version 7.0 (GraphPad Software, La Jolla, CA, U.S.A.). Moreover, the Student’s *t* test and one-way analysis of variance was employed for data comparison. A *P*-value <0.05 was regarded as a significant statistical difference.

## Results

### LSZ inhibited viability and proliferation of SK-OV-3 and OVCAR-3 cells

We first examined the effects of LSZ on the viability and proliferation ability of SK-OV-3 and OVCAR-3 cells by CCK-8 and colony formation assays. LSZ treatment markedly inhibited the viability of the cells (at 24 and 48 h, Figure 1A, *P*<0.05 and *P*<0.01, respectively) and the potential for cell proliferation (Figure 1B, *P*<0.01) of SK-OV-3 and OVCAR-3 cells in a dose-dependent manner. The intermediate concentration of 1 mM LSZ was used for the subsequent experiments.

**Figure 1:** Cell viability and proliferation ability following treatment with different concentrations of LSZ SK-OV-3 and OVCAR-3 cells were treated with different concentrations of LSZ and the cell viability (**A**) and proliferation (**B**) were evaluated by CCK-8 and colony formation assays, respectively, after incubation. *P<0.05, **P<0.01, ***P<0.001.

### LSZ inhibited migration and invasion of SK-OV-3 and OVCAR-3 cells

We further examined the effects of LSZ on the migration and invasion ability of SK-OV-3 and OVCAR-3 cells by scratch and transwell assays. As Figure 2 shows, LSZ treatment markedly inhibited the migration and invasion ability of SK-OV-3 and OVCAR-3 cells in a dose-dependent manner (*P*<0.01).

The article "Ligustrazine inhibits the proliferation and migration of ovarian cancer cells via regulating miR-211" was retracted in 2024. Reasons: plagiarized images; overlap with other authors' work; signs of a paper mill; concerns about the images.

**Figure 2:** Cell migration and invasion ability following treatment with different concentrations of LSZ SK-OV-3 and OVCAR-3 cells were treated with different concentrations of LSZ and the migration (**A**) and invasion (**B**) were evaluated by wound healing scratch and transwell assays, respectively, after incubation. *P<0.05, **P<0.01, ***P<0.001.

### LSZ increased the expression of miR-211 in SK-OV-3 and OVCAR-3 cells

The expression of miR-211 was significantly increased in SK-OV-3 and OVCAR-3 cells following treatment with LSZ (Figure 3A,B). Thus, we explored whether miR-211 expression could be regulated by the presence miR-211 inhibitors in 1 mM LSZ-treated SK-OV-3 cells. As shown in Figure 3C, 48 h after transfection, miR-211 inhibitors markedly decreased the levels of miR-211 in SK-OV-3 cells in comparison with the miR-211 negative control (NC)-treated cells, suggesting that transfection had been successfully performed; moreover, in the LSZ+miR-211 inhibitor treatment group, the level of miR-211 significantly decreased compared with LSZ treatment alone (Figure 3D, *P*<0.01).

**Figure 3:** Increased expression of miR-211 by LSZ Expression of miR-211 in SK-OV-3 (**A**) and OVCAR-3 (**B**) cells exposed to different concentrations of LSZ was evaluated by qRT-PCR. (**C**) Effects of miR-211 inhibitor on the expression of miR-211 in SK-OV-3 cells. (**D**) Effects of miR-211 inhibitor on the expression of miR-211 in LSZ-treated SK-OV-3 cells. *P<0.05, **P<0.01, ***P<0.001. Expression of miR-211 was normalized to the expression of U6.

### LSZ inhibited viability of SK-OV-3 cells by regulating the expression of miR-211

Next, the effects of miR-211 on the viability and proliferation of LSZ-treated SK-OV-3 cells were determined using the CCK-8 cell viability and colony formation assays. We found that the miR-211 inhibitor partially abrogated the LSZ-induced anti-tumor effects by increasing the cell viability and proliferation ability of LSZ-treated SK-OV-3 cells (Figure 4, *P*<0.01).

**Figure 4:** Inhibition of cell viability and proliferation by LSZ by regulating miR-211 expression Cell viability was determined using the CCK-8 (**A**) and colony formation (**B**) assay after exposure to different treatments. *P<0.05, **P<0.01, ***P<0.001.

### LSZ inhibited migration and invasion ability of SK-OV-3 cells by regulating the expression of miR-211

The effects of miR-211 on the migration and invasion ability of LSZ-treated SK-OV-3 cells were determined using the wound healing assay and transwell assay. As shown in Figure 5, LSZ significantly inhibited the migration (Figure 5A) and invasion (Figure 5B) of SK-OV-3 cells, and the transfection of miR-211 inhibitor led to increased migration of LSZ-treated SK-OV-3 cells (*P*<0.01).

The article "Ligustrazine inhibits the proliferation and migration of ovarian cancer cells via regulating miR-211" was retracted in 2024. Reasons: plagiarized images; overlap with other authors' work; signs of a paper mill; concerns about the images.

**Figure 5:** Inhibition of cell migration and invasion ability by LSZ by regulating miR-211 expression (**A**) The cell migration was determined by the wound healing assay after different treatments. (**B**) The cell invasion was determined by the transwell assay after different treatments. *P<0.05, **P<0.01.

### LSZ inhibited EMT of SK-OV-3 cells by regulating the expression of miR-211

Finally, the effects of miR-211 on the EMT of LSZ treated SK-OV-3 cells were examined. The expression of EMT markers was examined by the Western blotting assay. LSZ increased the expression of the epithelial markers E-cadherin and β-catenin and decreased the expression of the mesenchymal markers N-cadherin and vimentin. Conversely, transfection of the miR-211 inhibitor partially blocked the LSZ-induced anti-EMT effects by increasing the expression of E-cadherin and, and decreasing the expression of N-cadherin and vimentin in SK-OV-3 cells (Figure 6).

**Figure 6:** Inhibition of EMT by LSZ by regulating miR-211 expression The EMT of the cells was determined by Western blotting after different treatments.

## Discussion

In the present study, we evaluated the tumor suppressive roles of LSZ in an *in vitro* model of OC and investigated the related mechanism involved. We found that LSZ inhibited the proliferation, migration, invasion, and EMT of the OC cell line SK-OV-3 cells by regulating the expression of miR-211.

The tumor suppressive roles of LSZ have been discussed in several previous studies [10,11,27]. Yin et al. suggested that LSZ inhibits both migration and invasion [28], but not the numbers of SK-OV-3 and OVCAR-3 cells after a 24-h treatment. In the present study, we found that LSZ decreased the migration ability of SK-OV-3 cells at 24 h in a dose-dependent manner, which was consistent with the observation by Yin et al. [28]. Moreover, we also observed that LSZ did not exert a significant effect on the viability of SK-OV-3 and OVCAR-3 cells at 24 h, which was also consistent with Yin et al.’s findings, although when the culture time was extended to 48 h, we found that LSZ decreased the cell viability in a dose-dependent manner [28]. The above results suggested that LSZ inhibited the oncogenic behavior of OC cells *in vitro*. However, the underlying mechanism still requires further investigation.

The article "Ligustrazine inhibits the proliferation and migration of ovarian cancer cells via regulating miR-211" was retracted in 2024. Reasons: plagiarized images; overlap with other authors' work; signs of a paper mill; concerns about the images.

LSZ has been reported to affect the expression of miRNAs in different cell contexts in order to exert its biological activity. MiR-211 is considered a tumor suppressor in OC [27], and our finds show that miR-211 was up-regulated in LSZ-treated SK-OV-3 cells, and more importantly, transfection of a miR-211 inhibitor in LSZ-treated SK-OV-3 cells partially blocked the anti-tumor behavior of LSZ by increasing the viability, proliferation, and migration of the cells. Taken together, these results demonstrated the involvement of miR-211 in LSZ-induced anti-tumor effects, suggesting that LSZ may inhibit the growth and metastatic potential of OC cells by increasing the expression of miR-211.

EMT is considered an important cellular event during the progression of tumor metastasis [20,23]. It has been reported that LSZ could inhibit EMT in different types of cancer cells. Furthermore, miR-211 has also been found to inhibit the EMT of tumor cells. In our study, we found that LSZ increased the expression of the epithelial marker E-cadherin and decreased the expression of the mesenchymal markers N-cadherin and vimentin. Conversely, transfection of miR-211 inhibitor partially blocked LSZ-induced anti-EMT effects by increasing the expression of E-cadherin and decreasing the expression of N-cadherin and vimentin in SK-OV-3 cells. Our results suggested that LSZ inhibits the EMT of SK-OV-3 cells by regulating the expression of miR-211.

In conclusion, the present study revealed that LSZ may function as a tumor suppressor in OC; LSZ may exert its anti-tumor activity by increasing the expression of miR-211. Although further clinical and *in vivo* animal studies are still required to strengthen our conclusion, the present study may provide the theoretical basis for the potential application of LSZ as an alternative therapeutic strategy for the treatment of OC.

## Data Availability

The datasets used and/or analyzed during the current study are available from the corresponding author on reasonable request.

## Abbreviations

CCK-8: cell counting kit-8
EMT: epithelial–mesenchymal transition
GAPDH: glyceraldehyde-3-phosphate dehydrogenase
LSZ: Ligustrazine
miRNA: microRNA
miR-211: microRNA-211
M-MLV: moloney-murine leukemia virus
mRNA: messenger RNA
OC: ovarian cancer
